The article "The Hemodynamics of Patent Ductus Arteriosus in Patients after Central Shunt Operation" was published in 2021. Journal: Comput Math Methods Med.

# The Hemodynamics of Patent Ductus Arteriosus in Patients after Central Shunt Operation

**DOI:** 10.1155/2021/6675613

**Published:** 2021-04-24

**Authors:** Pan Xu, Haiyun Yuan, Jian Zhuang, Neichuan Zhang, Qianjun Jia, Yuhao Dong, Qifei Jian, Meiping Huang

**Affiliations:** ^1^School of Mechanical and Automotive Engineering, South China University of Technology, Guangzhou, 510640 Guangdong, China; ^2^Department of Cardiovascular Surgery, Guangdong Cardiovascular Institute, Guangdong Provincial Key Laboratory of South China Structural Heart Disease, Guangdong Provincial People's Hospital, Guangdong Academy of Medical Sciences, Guangzhou, China; ^3^Department of Catheterization Lab, Guangdong Cardiovascular Institute, Guangdong Provincial Key Laboratory of South China Structural Heart Disease, Guangdong Provincial People's Hospital, Guangdong Academy of Medical Sciences, Guangzhou, China

## Abstract

A central shunt (CS) was an important surgery of systemic-to-pulmonary shunt (SPS) for the treatment of complex congenital heart diseases with decreased pulmonary blood flow (CCHDs-DPBF). There was no clear conclusion on how to deal with unclosed patent ductus arteriosus (PDA) during CS surgery. This study expanded the knowledge base on PDA by exploring the influence of the closing process of the PDA on the hemodynamic parameters for the CS model. The initial three-dimensional (3D) geometry was reconstructed based on the patient's computed tomography (CT) data. Then, a CS configuration with three typical pulmonary artery (PA) dysplasia structures and different sizes of PDA was established. The three-element windkessel (3WK) multiscale coupling model was used to define boundary conditions for transient simulation through computational fluid dynamics (CFD). The results showed that the larger size of PDA led to a greater systemic-to-pulmonary shunt ratio (*Q*_S/A_), and the flow ratio of the left pulmonary artery (LPA) to right pulmonary artery (RPA) (*Q*_L/R_) was more close to 1, while both the proportion of high wall shear stress (WSS) areas and power loss decreased. The case of PDA nonclosure demonstrates that the aortic oxygen saturation (Sao_2_) increased, while the systemic oxygen delivery (Do_2_) decreased. In general, for the CS model with three typical PA dysplasia, the changing trends of hemodynamic parameters during the spontaneous closing process of PDA were roughly identical, and nonclosure of PDA had a series of hemodynamic advantages, but a larger PDA may cause excessive PA perfusion and was not conducive to reducing cyanosis symptoms.

## 1. Introduction

For infants with congenital heart disease and insufficient pulmonary blood flow, the systemic-to-pulmonary shunt (SPS) is the most commonly used clinical palliative surgical method, which mainly includes modified the Blalock-Taussig shunt (MBTS) and central shunt (CS) [1, 2]. Among them, CS surgery is establishing an artificial shunt between the ascending aorta (AAO) and the pulmonary artery (PA) to prompt the aortic blood flow into the pulmonary circulation [3]. As a vascular structure that connects the PA and the proximal descending aorta, the patent ductus arteriosus (PDA) is closely related to the effect of SPS surgery due to it being used as a spare connection similar to CS, and the PDA will spontaneously close after birth for normal infants [4]. Currently, the morbidity and mortality of patients receiving SPS intervention are still at a relatively high level due to the failure of the shunt procedure caused by the stenosis of the shunt and thrombosis [5, 6]. The management of SPS surgery for specific patients needs further improvement, and a much-debated question is whether PDA should be closed during the SPS operation.

Alwi et al. [7] have initially demonstrated that PDA stenting is a feasible surgery and could replace SPS for neonates with duct-dependent pulmonary circulation, but it will aggravate the preexisting branch PA stenosis at the implantation site of PDA stenting in patients with tetralogy of Fallot. Several studies have compared the postoperative data of the PDA stenting and the SPS surgery for different infants and found that the PDA stenting group is associated with fewer complications, shorter stay in the intensive care unit, and better development of PA, but there was no significant difference in mortality between the two groups [8, 9]. These studies have shown that unclosed PDA has some benefits in the palliative treatment of patients with insufficient pulmonary blood flow, although the PDA stents may cause a series of problems. Without using PDA stenting, Zahorec et al. [10] found that there were lower rates of reinterventions and mortality in the case of PDA nonclosure during the MBTS procedure in the clinic, and Zhang et al. [11] explained this clinical result by using steady computational fluid dynamics (CFD) indicating that retaining the PDA nonclosure during MBTS operation will provide a better hemodynamic environment. However, nonclosure of PDA in the SPS may associate with pulmonary hyperperfusion, which will cause a series of bad effects [12]. In general, most of the previous studies are retrospective studies for whether the PDA should be closed, and there are few works on the use of CFD to study the hemodynamics of such problems. And due to the connection form of CS and MBTS being quite different, it is impossible to infer the hemodynamic effects of this situation based on previous studies on MBTS. Therefore, we studied the effect of whether the PDA is closed in the CS surgery and further discussed the correlation between various hemodynamic parameters and the diameter of PDA, which was not done in our previous studies. Also, we abandoned the previous steady simulation method, and the transient simulation can get more meaningful data [13].

This research began with an analysis of the clinic data from patients with preoperative PDA nonclosure and decreased pulmonary blood flow who were prepared to receive a CS palliative surgery. Considering the effects of different types of PA dysplasia, the three-dimensional (3D) model of CS with three typical PA structures was established based on the preoperative computed tomography (CT) data in the clinic, including CS models with left pulmonary artery (LPA) dysplasia, symmetrical PA dysplasia, and right pulmonary artery (RPA) dysplasia. Also, the process of PDA spontaneous closure was simplified to six different relative sizes of PDA. Eventually, the transient simulation results were calculated by the CFD solver, and the effects of PDA in CS with different PA dysplasia were analyzed through multiple hemodynamic parameters.

## 2. Materials and Methods

### 2.1. Patient's CT Data and 3D Model Construction

This study was based on a 12-day-old infant with pulmonary atresia and symmetrical PA dysplasia and nonclosure PDA. Due to insufficient pulmonary blood flow, the surgeon implemented the CS operation on this patient. We consciously selected this kind of clinically controversial case on how to deal with PDA as the research object. To study the hemodynamics of such patients, the initial 3D geometry was rebuilt with this patient's 138-slice CT image collected in preoperation. And to eliminate the influence of the complexity of the AAO inlet cross-sectional shape on the calculation process and results, the AAO inlet was simplified to a circle and made an appropriate extension in the axial direction. Then, a 3.5 mm CS configuration was created in the 3D model based on the choice in the clinical CS surgery. The original irregularly shaped PDA was discarded, and with the axis of the original rebuilt PDA, a circular tube with a size of 1.5*D*_CS_ (where *D*_CS_ indicates the diameter of CS) was created as the latest initial nonclosure PDA. Finally, the model of CS with symmetrical PA dysplasia is shown in Figure 1(a).

The previous research showed that the hemodynamic environment was greatly affected by different types of RPA and LPA structures [14]. Thus, we have made a statistical size of branch PA based on the preoperative CT data of 40 infants with nonclosure of PDA before SPS operation from 2011 to 2017 provided by Guangdong Provincial People's Hospital, and it was found that the diameter ratios of the branch PA on both sides for the majority of patients were around 1.5, except for infants with the symmetrical PA dysplasia. Consequently, the PA dysplasia model is represented by a simplified PA model with reduced diameter, and three typical PA structures were defined: the PA structure of the infant selected in this study was symmetrical dysplasia (*D*_RPA_ = 4 mm, *D*_LPA_ = 4 mm, where *D*_RPA_ and *D*_LPA_ indicate the diameters of the RPA and LPA, respectively); the PA structure with LPA dysplasia (*D*_RPA_ = 6 mm, *D*_LPA_ = 4 mm); and the PA structure with RPA dysplasia (*D*_RPA_ = 4 mm, *D*_LPA_ = 6 mm). The 3D geometry of LPA (RPA) dysplasia was created through adjusting the size of LPA (RPA) and unchanging the initial position of LPA (RPA), based on the model of symmetrical PA dysplasia. The reconstructed structures are exhibited in Figures 1(b) and 1(c).

There will be a flow competition relationship in the PA due to the shunt blood being provided by both the CS and the nonclosure PDA. To highlight the impact of this competitive flow on the hemodynamics of patients after surgery, and considering the PDA being spontaneously closed for the postoperative patients, the relative sizes (*α*) was used to define the size of PDA:

(1) $$\begin{array}{c} \alpha =\frac{D_{\text{PDA}}}{D_{\text{CS}}}\cdot 100\%, \end{array}$$

where *D*_PDA_ and *D*_CS_ indicate the diameters of the PDA and CS, respectively.

The spontaneously closing process of PDA was simplified to the process of PDA relative sizes (*α*) decreased from 150% to 0 in this study. For CS models with each typical PA structure, six different relative sizes of PDA were established to correspond with six different degrees of PDA closure: the initial PDA nonclosure (*α* = 150), PDA gradually closing (*α* = 125%, *α* = 100%, *α* = 75%, and *α* = 50%), and PDA completely closed (*α* = 0). This study discarded the model with the relative size of PDA being *α* = 25% due to the undersized PDA always bringing about lower mesh quality for the model and affecting the accuracy of the simulation. Taking the case of PA structures with symmetrical PA dysplasia as an example, the changing processes of the PDA gradually closing are demonstrated in Figure 2.

### 2.2. Mesh Convergence Analysis

The 3D reconstruction models with tetrahedral elements and triangular prisms just for the boundary-fitted prism layers were meshed. The results of Benim et al. [15] show that the Shear Stress Transport (SST) *k*-omega model can be better suited for the numerical simulation of the SPS. Therefore, the determination of grid size in this study was based on the SST model, and the SPS models were meshed with six types of global element sizes (0.8 mm, 0.7 mm, 0.6 mm, 0.5 mm, 0.4 mm, and 0.3 mm) to get the grid independence test. According to the test results, the power loss change less than 1% was taken as the evaluation standard, and the final selected global element size was 0.4 mm to reduce the cost of calculation. Additionally, the boundary-fitted prism layers were defined with the first layer size being 0.1 mm and increased by a height ratio of 1.15 and 5 layers in total. The value of wall *Y* plus was checked to ensure the mesh quality of the boundary-fitted prism layer. Finally, the above grid parameter settings were adopted in all models, and the mesh information for the model with symmetrical PA dysplasia and nonclosure of PDA is described in Figure 3.

### 2.3. Boundary Condition and Calculation Methods

In this study, a three-element windkessel (3WK) model consists of two resistors, and one capacitor was used to prescribe the outlet boundary conditions of the 3D vascular model [16], and the clinically measured aortic flow parameter was used as the inlet boundary condition of the 3D models. This 3WK multiscale coupling model is one of the most typical open-loop multiscale coupling models. In the calculation process, each iteration step will perform a coupling calculation of 0D and 3D. The average outlet pressure of the 3D model is calculated by the 0D model, and the outlet cross-sectional flow calculated by the 3D model is used as the condition for the iterative calculation of the 0D model. Marsden [17] shows that for patients who provide parameters such as aortic inlet flow in the clinical process, the open-loop multiscale coupling model can better ensure the stability and convergence of the simulation. In our study, the Doppler echocardiogram of the patient's aortic inlet in the resting state was collected and converted into a flow waveform. Therefore, this open-loop multiscale coupling model was selected for our simulation. For an example of the CS model with symmetrical PA dysplasia and nonclosure of PDA, the final 3WK multiscale coupling model diagram is shown in Figure 4, a flow waveform (as shown in Figure 4(b)) was applied at the inlet of the ascending aorta (AAO), and the six outlets (innominate artery (IA), left common carotid artery (LCA), left subclavian artery (LSA), descending aorta (DAO), LPA, and RPA) were coupled with the 3WK model.

According to the 3WK model shown in Figure 4(c) and using the method of integrating factors, the outlet pressure can be calculated as follows [18, 19]:

(2) $$\begin{array}{c} P\left(t\right)=R^{0}Q\left(t\right)+P^{0}\left(0\right)e^{-t/\left({CR}^{1}\right)}+\frac{e^{-t/\left({CR}^{1}\right)}}{C}\int_{0}^{t}\left(\frac{P^{d}}{R^{1}}+Q\left(t\right)\right)e^{t/\left({CR}^{1}\right)}dt, \end{array}$$

where *R*^0^ and *R*^1^ indicate the flow resistance at the proximal and distal ends, respectively; *P*^0^(0), *P*^*d*^, and *P*(*t*) are the proximal pressure, the downstream pressure, and the outlet pressure at the initial time, respectively; *C* represents the compliance of the blood vessel; and *Q*(*t*) is the outlet volume flow rate.

The 3WK model parameters *R*^0^, *R*^1^, and *C* in the case of the CS model with symmetrical PA dysplasia were calculated based on the clinical parameters and previous studies [20–22]. Since the CS model with RPA or LPA dysplasia has the same aortic structure, it is assumed that only the parameter values of the 3WK model of the PA outlets need to be adjusted, while these parameter values of the other outlets remain unchanged. Therefore, according to the previous study of Pietrabissa et al. [23], we have assumed that the value of characteristic resistance (*R*^0^) at each outlet is inversely proportional to the square of the cross-sectional area of the outlet and the compliance (*C*) value is proportional to the cube of the outlet radius; then, the 3WK parameters of the unilateral PA dysplasia model can be calculated based on the symmetrical PA dysplasia model. Finally, the pulse pressure method was used to calibrate the parameter values of the 3WK model [24, 25], and the determined parameter values for all models are shown in Table 1.

User-defined functions are used to customize outlet boundary conditions during the simulation, and considering the calculation accuracy and workload, the second-order Runge-Kutta method was used to discretize the integral term. According to the measurement data provided by Di Molfetta et al. [26], the simulation results of pulmonary pressure in this study were within a reasonable range.

All models have used the same calculation method; the blood was assumed to an incompressible Newtonian fluid, with the dynamic viscosity of 0.0035 Pa·s. And the density was 1060 kg/m^3^ [27, 28]. It is assumed that the blood vessel wall was rigid and impermeable [29]. Additionally, the *K*-omega based Shear Stress Transport (SST) solver was set as the turbulence calculation mode [15], and a second-order accurate numerical space discretization scheme was adopted for the 3D model. The residual values of the continuity, velocity component, turbulent kinetic energy, and omega were set to 10^−6^, and the total calculation time length is five cardiac cycles with 0.5 s for each cycle. Finally, the number of time steps in a single cardiac cycle was set to 1000, and transient CFD simulation was conducted to obtain the characteristics of the flow field.

### 2.4. Hemodynamic Parameters

The main purpose of CS surgery was to provide a certain amount of shunt blood for the pulmonary circulation through establishing an artificial shunt, which could increase the body's blood oxygen content and reduce the patient's cyanosis symptoms and promotes the development of the PA [30–32]. Therefore, a series of postoperative clinical evaluation parameters were analyzed in this study. Among them, the systemic-to-pulmonary shunt ratio (*Q*_S/A_) was usually used to express the volume flow of shunt blood:

(3) $$\begin{array}{c} Q_{\text{S}/\text{A}}=\frac{Q_{\text{shunt}}}{Q_{\text{AOO}}}, \end{array}$$

where *Q*_shunt_ and *Q*_AAO_ indicate the total volume flow in the pulmonary circulation and the inlet of AAO during a cardiac cycle, respectively.

Studies have confirmed that promoting the balanced distribution of pulmonary blood flow after CS surgery is crucially important [33]. Thus, the LPA/RPA flow ratio (*Q*_L/R_) was adopted to evaluate the patient's LPA and RPA perfusion after surgery:

(4) $$\begin{array}{c} Q_{\text{L}/\text{R}}=\frac{Q_{\text{LPA}}}{Q_{\text{RPA}}}, \end{array}$$

where *Q*_LPA_ and *Q*_RPA_ indicate the flow volume in the LPA and RPA within one cardiac cycle, respectively.

The power loss and the indexed power loss (iPL) are an important indicator for evaluating hemodynamics after CS surgery; especially for patients with poorly developed cardiac function, the excessive power loss will affect the patient's capacity to perform physical activities after surgery [34, 35]:

(5) $$\begin{array}{c} \text{PL}=\frac{1}{N}\overset{N}{\underset{\text{i}=1}{\sum }}\left(\underset{\text{in}}{\sum }\left(p+\frac{1}{2}\rho v^{2}\right)Q-\underset{\text{out}}{\sum }\left(p+\frac{1}{2}\rho v^{2}\right)Q\right),\\ \text{iPL}=\frac{\text{NPL}}{\sum_{i=1}^{N}\sum_{\text{in}}\left(p+1/2\rho v^{2}\right)}. \end{array}$$

Among them, *p* is the static pressure of the blood in the resting state, *ρ* is the density of the blood, *v* is the flow velocity of the blood at the border of the inlet and outlet of the 3D model, *Q* is the volume flow of the blood at the inlet and outlet of the 3D model, and *N* represents the total calculation time steps in a cardiac cycle.

The calculation of blood oxygen content after surgery is an important indicator for evaluating the central shunt, and it is closely related to whether the patient needs further intervention after surgery [36, 37]. According to the previous studies, the system oxygen delivery volume (Do_2_) and aortic oxygen saturation (Sao_2_) are as follows:

(6) $$\begin{array}{c} {\text{DO}}_{2}=Q_{\text{S}}C_{{\text{PVo}}_{2}}-\frac{Q_{\text{S}}}{Q_{\text{P}}}{\text{CVo}}_{2},\\ {\text{Sao}}_{2}=98-\frac{24}{{\text{Q}}_{\text{S}}}, \end{array}$$

where *Q*_S_ and *Q*_P_ indicate the volume flow into the systemic circulation and the volume flow into the pulmonary circulation, respectively. According to clinical statistics [38, 39], the oxygen saturation percentage of the pulmonary vein was set to 98% and the oxygen content (*C*_PVo_2__) flowing into the ventricle through the pulmonary circulation and the oxygen consumption (CVo_2_) of the body were 0.22 mLo_2_/mL and 0.874 mLo_2_/s, respectively.

## 3. Result

### 3.1. The Systemic-to-Pulmonary Shunt Ratio and the LPA/RPA Ratio

As detailed in Figure 5, there are noticeable differences in *Q*_S/A_ and *Q*_L/R_ of the three typical PA configuration models with the CS. With the relative sizes of PDA (*α*) decreased from 150 to 0, *Q*_S/A_ of the case with symmetrical PA dysplasia, LPA dysplasia, and RPA dysplasia gradually decreased from 0.73 to 0.56, 0.77 to 0.58, and 0.78 to 0.59, respectively. This analysis found that the nonclosure of PDA increases the *Q*_S/A_ value of the CS model, and the *Q*_S/A_ value will gradually decrease following the *α* decrease. In most cases, *Q*_L/R_ > 1, which indicates that more blood flow was in LPA than RPA. The only two exceptions were the cases of RPA dysplasia when *α* was 150 and 125; the corresponding value of *Q*_L/R_ was 0.97 and 0.94, respectively. A further novel finding was that the nonclosure of PDA was associated with lower *Q*_L/R_ than the closure of PDA.

### 3.2. Power Loss and Indexed Power Loss

Figure 6 depicts the variation of power loss and iPL with the different relative sizes of PDA. For cases with nonclosure PDA (closure of PDA), the power loss of symmetrical PA dysplasia, LPA dysplasia, and RPA dysplasia models was 182 mW (288 mW), 170 mW (283 mW), and 166 mW (282 mW), respectively. The evidence suggests that the power loss and iPL of the CS model were increased monotonically with the relative sizes of the PDA decreases; the lower value of iPL was beneficial to the postoperative recovery.

### 3.3. Systemic Oxygen Delivery and Aortic Oxygen Saturation

For the three typical PA configuration models with the CS, the changes of the Do_2_ and the Sao_2_ when the PDA was gradually closed are shown in Figure 7. The simulation results demonstrated that the Do_2_ of the symmetrical PA dysplasia, the LPA dysplasia, and the RPA dysplasia models with the nonclosure of PDA (closure of PDA) was 2.19 mLo_2_/s (3.45 mLo_2_/s), 1.83 mLo_2_/s (3.38 mLo_2_/s), and 1.98 mLo_2_/s (3.09 mLo_2_/s), respectively. It appears that with the gradual atresia of PDA, Sao_2_ will gradually decrease while the Do_2_ gradually increases, which has opposite effects for the patients.

### 3.4. WSS Distribution and 3D Blood Flow Streamlines

According to the research of Holme et al. [40] and Maalej and Folts [41], the low WSS range is defined as 0-50 Pa, and the medium WSS range that can cause platelet-mediated activation is 50-140 Pa; the range of high WSS that can lead to platelet-mediated thrombosis is greater than 140 Pa. In this study, the blood flow during systole (*t* = 0.12 s) was selected as the research object. The proportion of different WSS distribution was plotted for the CS configuration with the three typical PA structures (as shown in Figures 8(a), 9(a), and 10(a)). For the cases of nonclosure PDA (closure PDA), the proportion of the medium WSS areas and high WSS areas in total areas of the symmetrical PA dysplasia model is 18.6% and 0.9% (18.2% and 3.1%), while the LPA dysplasia model is 16.8% and 1.1% (17.7% and 2.9%), and the RPA dysplasia model is 17.1% and 1.1% (16.8% and 3.2%), respectively. Obviously, the nonclosure of PDA will decrease the areas of high WSS by more than 60% and slightly change in the medium WSS areas. It is worth noting that the closure of PDA may decrease the area of high WSS compared to the case where the relative size of the PDA is *α* = 50. From Figures 8(b), 9(b), and 10(b), it is clear that the high WSS areas distribute near the anastomosis of the central shunt to the AAO and PA when the PDA was closed, while the high WSS areas at the corresponding position are significantly reduced when the PDA was nonclosure. Furthermore, the 3D blood flow streamlines show a higher velocity of corresponding blood flow in the CS when *α* = 0, while the complex flow phenomenon presents at the PA when *α* = 150% (Figures 8(c), 9(c), and 10(c)). Compared with the symmetrical PA dysplasia and LPA dysplasia configuration models, the nonclosure of PDA has a fewer effect on the flow velocity of the RPA dysplasia configuration model.

## 4. Discussion

For the CS model with different PA structures and nonclosure of PDA in preoperation, we have studied the hemodynamic changes during the closing process of PDA. The simulation results show that the nonclosure of PDA in CS surgery may associate with a better hemodynamic environment, which is similar to the result of the previous study for PDA management during the MBTS [11]. Our study expanded the knowledge base on PDA by exploring the influence of the closing process of the PDA on the hemodynamic parameters for the CS model with three typical structures of the PA dysplasia.

Compared with the CS model when the PDA is in the atretic state, the nonclosure PDA is equivalent to providing an additional shunt channel from the systemic circulation to the pulmonary circulation. These results demonstrated that under the shunt diameter of 3.5 mm, CS has been able to provide sufficient PA perfusion for the research subjects when the PDA was closed. However, the presence of PDA led to an increase in the *Q*_S/A_ value and PA perfusion of the CS model, which may accompany the risk of heart failure and pulmonary hypertension caused by excessive PA perfusion [12]. Thus, for patients with a higher risk of PA overflow, it is not recommended to keep a larger size of PDA. It is worth noting that the *Q*_S/A_ value has decreased very gently when the PDA size is smaller (*α* < 50), which indicated that this size of PDA has less impact on the risk of PA overflow. Moreover, *Q*_S/A_ is closely related to Do_2_ and Sao_2_. The cyanosis phenomenon in patients becomes alleviated with the increase of Do_2_ and Sao_2_, which is the main purpose of SPS surgery. However, the nonclosure of PDA may cause a lower Do_2_ and higher Sao_2_ in our study due to the overlarge *Q*_S/A_ causing too little blood involved in the systemic circulation. Such results are beneficial to the development of PA, but not conducive to reducing the cyanosis phenomenon.

The CS structure and PA have a strong geometric sensitivity, which may cause asymmetrical blood flow distribution in the LPA and RPA when the PDA was closed. And this result will be improved in the case of PDA nonclosure; especially for the models with symmetrical PA dysplasia or LPA dysplasia in the PDA nonclosure states, *Q*_L/R_ is close to 1, which is the infusive result and could promote the balanced development of LPA and RPA. For the model with RPA dysplasia, the case of PDA closure with *Q*_L/R_ = 5.22 indicates that CS is not suitable for this patient, and combined with the research of Mitra and McNamara [12], MBTS could be considered a better choice at this time. However, the results demonstrate that the *Q*_L/R_ value is reduced to 2.06 similar to the MBTS in the PDA nonclosure. Therefore, for the case of PDA nonclosure, CS will lead to more uniform pulmonary blood flow distribution than BT. In general, if promoting the balanced development of the LPA and RPA after CS surgery is the most important goal, a PDA that remains in the conductive state can be the first choice.

Our study demonstrates that nonclosure of PDA tends to result in lower power loss and iPL of the CS model with three typical PA dysplasia structures, and retaining the initial PDA reduces the power loss of the CS model by more than 30% compared with the PDA closed. The value of power loss and iPL is negatively correlated with PDA size, while the structural difference of PA has little effect on this changing trend. Lower power loss is beneficial to reduce the burden on the heart of patients with hypoplastic cardiac function and provide patients with a better quality of life in postoperation [42]. This implies that PDA nonclosure during the surgery is beneficial for patients to recover in the postoperation before PDA is closed spontaneously. Thus, surgeons could consider retaining the PDA when myocardial dysplasia is a major problem for the patients.

The unclosed PDA is considered an additional shunt pipe, which can greatly reduce the probability of complete blockage of the systemic-to-pulmonary shunt and plays a positive role in preventing SPS failure caused by early acute shunt thrombosis. From the result, the case of PDA nonclosure has shown the homogeneous WSS distribution and the smaller proportion of high WSS areas. The high WSS will mediate the activation of platelets, and in the area of low flow rate, the activated platelets will aggregate and combine with the coagulation protein in the low blood flow areas, which is a precursor to thrombosis [41]. Therefore, it is preferable to keep the PDA in the conductive state to reduce the risk of thrombosis in the CS after surgery. Moreover, it should be noted that when the relative size of the PDA is too small (*α* < 50), keeping the PDA nonclosure may increase the risk of shunt blockage. It is recommended to manually turn off PDA in CS operation when *α* is smaller than 50.

The shunt blood for pulmonary circulation provided by the CS and the PDA are mixed in the PA, which resulted in a complicated blood flow pattern at the junction, while the blood velocity distribution of the CS structure is more uniform. In addition, the surgeon cannot ignore the changes in hemodynamic parameters during the process of PDA spontaneously closed and how to deal with different sizes of PDA before surgery. Our results clearly show that the power loss, RPL, and Do_2_ are negatively correlated with the relative size of PDA, while Sao_2_ is positively correlated with it, which is consistent with the result of MBTS with nonclosure of PDA in Zhang et al.'s study [11].

This study focuses on the influence of the diameter of PDA and PA on hemodynamics, and the diameter of blood vessels may be one of the most important factors affecting hemodynamics [43]. However, there were still some limitations in our conclusion. For example, our statistics on PA dysplasia are only based on a single database of the local hospital. And the geometric diversity of PA, aorta, and PDA in different patients may affect hemodynamics. This requires us to do more extensive statistics and research in the future. Moreover, the geometry of the CS anastomosis is simplified; this factor will also have an impact on the simulation results [44]. Besides, regarding the influence of PDA spontaneous closure on postoperative CS, we are currently only simulating and analyzing based on a fixed CFD model. On the one hand, it is necessary to verify the accuracy of the CFD simulation results through a postoperative follow-up; on the other hand, as the patient grows after surgery, the size of the cardiovascular structure may slowly grow, which may cause the original simulation model to be no longer accurate.

## 5. Conclusion

For the CS model with symmetrical PA dysplasia, LPA dysplasia, and RPA dysplasia, respectively, the changing trends of hemodynamic parameters during the spontaneous closing process of PDA were roughly identical. Nonclosure of PDA has a series of advantages, which could provide more uniform pulmonary blood flow to promote the balanced development of LPA and RPA, as well as reduce power loss to decrease the heart workload and reduce the proportion of high WSS areas to prevent postoperative shunt thrombosis. Besides, the dual shunt is beneficial in preventing early acute shunt failure. However, the gradual closure of PDA will make these advantages nonexistent. It is worth noting that the systemic-to-pulmonary shunt ratio (*Q*_S/A_) of CS surgery is positively correlated with the size of PDA, and a larger PDA may cause excessive PA perfusion and is not conducive to increasing oxygen delivery to reduce cyanosis symptoms. Moreover, it cannot be ignored that different PA structures have obvious effects on *Q*_S/A_, *Q*_L/R_, and oxygen transfer. There is no gold standard for how to manage PDA during CS surgery, the specificity of the cardiovascular geometry and physical condition in different patients limits the application scope of our research results, and multiple hemodynamic parameters should be considered comprehensively according to the characteristics of different patients to achieve the best surgical effect.

## Figures and Tables

**Figure 1:** Model of CS with nonclosure of PDA in three typical PA structures: the symmetrical PA dysplasia (*D*_RPA_ = 4 mm, *D*_LPA_ = 4 mm), the LPA dysplasia (*D*_RPA_ = 6 mm, *D*_LPA_ = 4 mm), and the RPA dysplasia (*D*_RPA_ = 4 mm, *D*_LPA_ = 6 mm).

**Figure 2:** The 3D reconstruction geometry of the PDA closing process: the initial arterial structure (*α* = 150%), the arterial structure during PDA closing (*α* = 125%, *α* = 100%, *α* = 75%, and *α* = 50%), and PDA completely closed (*α* = 0).

**Figure 3:** The information of mesh for the model with symmetrical PA dysplasia and nonclosure of PDA.

**Figure 4:** Schematic of the 3WK multiscale coupling model for the case of the CS model with symmetrical PA dysplasia and nonclosure of PDA.

**Figure 5:** The changing process of the systemic-to-pulmonary shunt ratio (*Q*_S/A_) and the LPA/RPA ratio (*Q*_L/R_) with different relative sizes of PDA (*α*).

**Figure 6:** Power loss (PL) and indexed power loss (iPL) with the different relative sizes of PDA (*α*).

**Figure 7:** Effect of PDA size on systemic oxygen delivery (Do_2_) and aortic oxygen saturation (Sao_2_) for three typical PA configurations.

**Figure 8:** The WSS distribution and 3D blood flow streamline for the case of the symmetrical PA dysplasia model.

**Figure 9:** The WSS distribution and 3D blood flow streamline for the case of the LPA dysplasia model.

**Figure 10:** The WSS distribution and 3D blood flow streamline for the case of the RPA dysplasia model.

**Table 1:** Resistance and capacitance parameter values of the 3WK model under three typical PA structures: (a) the symmetrical PA dysplasia, (b) the LPA dysplasia, and (c) the RPA dysplasia.

Outlet boundary	*R* ^0^ (Pa s/mL)	*R* ^1^ (Pa s/mL)	*C* (mL/Pa)
IA	55.3	1817	0.001644
LCA	118	3627	0.00077
LSA	97	3678	0.000934
DAO	18.8	1025	0.000482
LPA(a)	166.7	4.3	0.0034814
RPA(a)	166.7	4.3	0.0034814
LPA(b)	166.7	4.3	0.0034814
RPA(b)	41.7	1.07	0.01044
LPA(c)	41.7	1.07	0.01044
RPA(c)	166.7	4.3	0.0034814

## Data Availability

The data used to support the findings of this study are available from the corresponding authors upon request.
